# Mechanism of Emodin in the Treatment of Rheumatoid Arthritis

**DOI:** 10.1155/2022/9482570

**Published:** 2022-10-03

**Authors:** Lianying Cheng, Jie Chen, Xiaofeng Rong

**Affiliations:** ^1^Department of Combination of Chinese and Western Medicine, The First Affiliated Hospital of Chongqing Medical University, Chongqing 400016, China; ^2^Department of Orthopedics, The First Affiliated Hospital of Chongqing Medical University, Chongqing 400016, China

## Abstract

Rheumatoid arthritis (RA) is a chronic, systemic, and autoimmune disease, and its main pathological changes are inflammatory cell infiltration accompanied by the secretion and accumulation of a variety of related cytokines, which induce the destruction of cartilage and bone tissue. Therefore, the modulation of inflammatory cells and cytokines is a key therapeutic target for controlling inflammation in RA. This review details the effects of emodin on the differentiation and maturation of T lymphocytes, dendritic cells, and regulatory T cells. In addition, the systematic introduction of emodin directly or indirectly affects proinflammatory cytokines (TNF-*α*, IL-6, IL-1, IL-1*β*, IL-17, IL-19, and M-CSF) and anti-inflammatory cytokines (the secretion of IL-4, IL-10, IL-13, and TGF-*β*) through the coregulation of a variety of inflammatory cytokines to inhibit inflammation in RA and promote recovery. Understanding the potential mechanism of emodin in the treatment of RA in detail provides a systematic theoretical basis for the clinical application of emodin in the future.

## 1. Introduction

Rheumatoid arthritis (RA) is an autoimmune disease characterized by chronic and erosive arthritis with an incidence of 0.5–1% worldwide, and its pathological changes are chronic inflammation of the joint synovium and pannus formation [1–3]. RA not only is accompanied by progressive joint damage but also involves cardiovascular, lung, kidney, and multiple organ damage. Additionally, RA can lead to multiple rheumatic immune diseases, such as systemic lupus erythematosus, and declines in participation in social activities and quality of life. Furthermore, long-term medical treatment can increase the psychological burden of patients and even lead to mental illnesses such as depression [3, 4]. The pathogenesis of RA is unclear, and some studies have shown that RA pathogenesis is related to abnormal immune responses mediated by antigens (foreign or self), antigen-presenting cells, lymphocytes, and cytokines [1, 5, 6] In RA, inflammation is an important factor leading to disease progression, and inflammatory cytokines play an important role. Inflammatory cytokines include proinflammatory and anti-inflammatory cytokines. Proinflammatory cytokines include tumor necrosis factor (TNF)-ɑ, IL-6, IL-1, IL-1*β*, IL-17, IL-9, and M-CSF, which play key regulatory roles in cell proliferation, apoptosis, and innate and adaptive immunity. In addition, anti-inflammatory cytokines, including IL-4, IL-10, IL-13, and transforming growth factor-*β* (TGF-*β*), can balance the chronic activation of innate and adaptive immune cells [7, 8]. The treatment of RA is mainly based on targeting inflammatory cytokine receptors with biological agents and disease-modifying antirheumatic drugs (DMARDs). A TNF inhibitor (TNFi) that inhibits inflammation prior to RA is effective and popular in the clinic, but its long-term use can induce drug dependence and side effects. Research has shown that traditional Chinese medicine has great potential for the treatment of RA. In particular, emodin can effectively balance the levels of proinflammatory and anti-inflammatory cytokines to treat RA and thus prevent the adverse effects of targeting a single regulatory mechanism. Therefore, this article reviews the effect of emodin on the disease process of RA through the regulation of inflammatory cytokines.

## 2. Basic Biology of Emodin

The traditional Chinese medicine(TCM) RHEI RADIX ET RHIZOMA (Figure 1(a)) is called “Commander”, was first recorded in the classic book “Shennong's Herbal Classic” and was used clinically approximately 2,000 years ago in China. This representative TCM laxative can be used to treat coagulated cold by purgation, clearing heat-fire, eliminating blood stasis by catharsis, cooling the blood to resolve macula, clearing heat, and promoting diuresis [9, 10]. Modern research shows that Rt exerts good anti-inflammatory and antitumor effects and can regulate intestinal flora [11–13]. The main component of Rt is the anthraquinone, which can be further separated into free anthraquinone and conjugated anthraquinones, such as emodin, aloe-emodin, rhein, chrysophanol, and emodin methyl ether [14]. Emodin (chemical name: 1′3′8-trihydroxy-6-methylanthraquinone; molecular weight: 270.24) (Figure 1(b)) is a class of biologically active natural products that has recently received much attention. Emodin has a variety of biological regulatory functions, such as immunosuppression and antitumor, antioxidant and anti-inflammatory activities (Figure 1(c)). Therefore, emodin has therapeutic potential in diseases of the cardiovascular system, respiratory system, metabolic system, nervous system, and other systems.

### 2.1. Pharmacokinetics of Emodin

The main metabolic pathway of emodin is glucuronidation metabolism, followed by sulfonation metabolism [15]. Emodin exists in the plasma, kidney, and lung as glucuronide or sulfate ester and in the liver as emodin in free form [16]. The absorption, excretion, tissue distribution, and metabolism of [I4C] emodin have been studied in rats after a single oral administration (approximately 50 mg/kg). An analysis of the urine revealed excretion of 18% of the administered dose within 24 h and 22% of the administered dose within 72 h. The metabolites excreted in urine were mainly free anthraquinone, and the content of glucuronide or sulfate was only approximately 3%. At 24–120 h, the emodin detected in feces was mainly free, and the level equaled 48% or 68% of the administered dose. At 3–5 d, radioactivity was significantly reduced in most organs; however, high radioactivity remained in the kidneys until 5 d. At 72–120 h, radioactivity was greatly increased in mesenteric and adipose tissue [17]. An analysis of the half-life of emodin in rabbits revealed that its metabolic process in vivo involved a two-compartment open model. The AUC of emodin was 518 *μ*g·min/mL, the clearance was 72.3 ml/min, and the elimination half-life was 227 min. The protein binding of emodin was investigated by the equilibrium dialysis method. Emodin was found to be highly bound (99.6%) to serum protein [18].

In vivo and in vitro experimental studies predicted that the target organs of emodin in which toxicity can occur are the kidney and liver [19], which may interfere with glutathione and fatty acid metabolism in human hepatocytes [20] and induce renal tubular pigmentation in male and female mice and an increase in the incidence of kidney disease in female mice. Moreover, emodin is reproductively toxic and inhibits human sperm function by reducing the sperm [Ca2+] i and inhibiting tyrosine phosphorylation in vitro [21].

### 2.2. Use of Emodin to Treat Human Diseases

Emodin has potential therapeutic effects on various diseases (Figure 2). Emodin can inhibit the proliferation and angiogenesis of tumor cells, reduce drug resistance and improve chemotherapy sensitivity in tumors and has a wide range of therapeutic effects on lung cancer, pancreatic cancer, breast cancer, and other tumors [22–25]. In metabolic disease, emodin improves dysglycemia and metabolic disorders in diabetes patients by inhibiting the activity of 11*β*-hydroxysteroid dehydrogenase type 1 inhibitor in adipose tissue [26], and in oral diseases, emodin reduces the nitric oxide (NO) levels in peripheral blood and gingival tissue and inhibits inflammatory responses and alveolar bone resorption [27]. In liver diseases, emodin can improve ethanol-mediated hepatic steatosis and treat alcoholic liver disease by downregulating the levels of alanine aminotransferase (ALT), triglyceride, and aspartate aminotransferase [28]. In microbial regulation, emodin can promote the expression of related resistance genes in host cells, destroy microbial cell membranes and inhibit the replication of microbial DNA to effectively suppress the replication of pathogenic microorganisms and damage host cells [29–33]. Regarding oxidative stress damage, emodin exerts potential antioxidant effects, such as regulating the free radical and reactive oxygen species (ROS) levels and affecting oxidative stress-induced damage [34]. In cardiovascular diseases, emodin exerts potential therapeutic effects on diabetic retinopathy by inhibiting aldose reductase activity and improving retinal angiogenesis [35]. Emodin can also significantly inhibit the expression of TNF-*α* and activate the NF-*κ*B signaling pathway in the local myocardial infarction area and can play a protective role in myocardial ischemia [36]. In respiratory diseases, emodin can effectively reduce pulmonary inflammatory cell infiltration, mucus secretion and serum IgE production, and regulate lung injury through IL-4-mediated macrophage polarization, STAT6 phosphorylation, and Nrf2 antioxidant signaling pathway activation [37, 38]. In neurological diseases, emodin directly protects nerve cells by regulating hormones, nerve growth factor (NGF), and related signaling pathways [39]. In immunomodulation, emodin can directly regulate the activity of immune cells or regulate related proinflammatory or anti-inflammatory cytokines secreted by immune cells and thereby regulate the inflammatory damage induced by immune disorders [40].

### 2.3. Regulation of Emodin in Immune Cells

The immunoregulatory function of emodin mainly affects the differentiation and maturation of T lymphocytes, dendritic cells (DCs), and regulatory T cells (Tregs) and the secretion of a variety of proinflammatory and anti-inflammatory cytokines to achieve immunomodulatory effects (Figure 3) [41].

T lymphocytes are also known as T cells and originate from bone marrow-derived lymphoid stem cells. T cells mainly include helper T (Th) cells (CD4^+^ cells), effector T (Te) cells, cytotoxic T (Tc) cells, virgin or natural T cells, and memory T (Tm) cells. CD4^+^ T cells are further classified as Th1, Th2, Th17, Treg, and Tfh cells and play important roles in cellular immunity. Th1 cells can secrete the cytokines IFN-*γ*, IL-2, and TNF-*α*; as a result, Th1 cells, thus mediate the activation of macrophages through IFN-*γ* and the proliferation of CD8^+^ T cells through IL-2, induce B cells to differentiate immunoglobulins, promote complement fixation and delayed-type hypersensitivity and aid in intracellular microbial clearance [42, 43]. Th2 cells can secrete IL-3, IL-4, IL-5, IL-10, and IL-13, and these cells can thereby mediate B-cell differentiation through IL-4, participate in allergic reactions and mediate macrophage deactivation through IL-4, IL-10 and IL-13 [44, 45]. Th17 cells can secrete the cytokines IL-17A, IL-17F, IL-22, and TNF-*α* and can mobilize and activate neutrophils through secreted IL-17 A/F, and these cells thereby induce autoimmune responses, tumor inflammatory responses, or transplant immune rejection [46]. Tregs can secrete the regulatory factor forkhead box protein 3 (Foxp3) and the cytokines IL-4, IL-10, and TGF-*β*, which can inhibit the proliferation and activation of T cells through secreted IL-10 and TGF-*β*, and these cells, thus exert immunosuppressive effects and regulate autoimmune tolerance [47, 48]. Tfh cells can secrete the cytokines Bcl-6, IL-21, CXCR5, and ICOS, participate in information transmission during B-cell differentiation, aid the activation of B cells, promote the formation of germinal centers and the secretion of immunoglobulins, and maintain the long-term immune response [49, 50].

DCs originate from bone marrow pluripotent hematopoietic stem cells [51, 52], are the most powerful professional antigen-presenting cells (APCs) in the body and can efficiently take up, process, and present antigens [51]. DCs can induce the production of specific cytotoxic T lymphocytes (CTLs). The combination of DCs with T cells can result in high levels of IL-12 and IL-18 secretion and thereby activate T-cell proliferation, induce CTL generation, and dominate Th1 immune responses. DCs promote NK-cell killing via perforin P and FasL/Fas. DCs can also secrete specific chemokines to attract and recruit T cells and ultimately activate the inflammatory response of T cells [45, 53].

Tregs, which are a T-cell subset that controls autoimmune responses in the body, can be divided into naturally occurring natural regulatory T cells (nTregs), induced adaptive regulatory T cells (iTregs), CD8^+^ Tregs, and NKT cells [54]. nTregs have not been shown to play an immunoregulatory role by secreting related cytokines. iTregs mainly include Tr1 and Th3 cells. Tr1 cells inhibit the proliferation of naïve and memory T cells by secreting IL-10 and TGF-*β*. Th3 cells can secrete a large amount of TGF-*β*, which has inhibitory effects on Th1 and Th2 cells. Th3 cells can secrete TGF-*β*, IL-4 and IL-10 after antigen-specific activation [55]. There are two subsets of CD8^+^ Tregs, CD28^+^ and CD28^−^, and CD8^+^CD28^−^ Tregs exert immunosuppressive effects [56]. Natural killer T cells (NKTs) are a unique group of *αβ* T cells that express the T-cell receptor (TCR*αβ*, b) and the NK-cell receptors NK1.1 or NK161. In addition, NKT cells can rapidly secrete a large amount of the Th2-type cytokines IL-4 and IL-10 and secrete IL-13 to regulate the function of CD8+ T cells, and these cells, thus, control the occurrence of various autoimmune diseases. In addition, NKT cells can enhance immune killing effects through the rapid secretion of IFN-r, TNF, and other Th1-type cytokines [57].

Emodin induces T-cell apoptosis in vitro through ROS-mediated endoplasmic reticulum stress and mitochondrial dysfunction, and previous studies have revealed elevated levels of intracellular free Ca2^+^ and intracytoplasmic cytochrome C, the activation of cleaved caspase-3, caspase-4, and caspase-9, and disruption of the mitochondrial membrane potential [40]. Emodin can inhibit the secretion of IFN-*γ* by T cells, reduce the numbers of CD3^+^CD4^+^IL4^+^, CD3^+^CD4^+^ IFN-*γ*^+^, CD3^+^CD8^+^IL4^+^, and CD3^+^CD8^+^ IFN-*γ*^+^ T cells among peripheral blood mononuclear cells and splenic lymphocytes and exert anti-inflammatory effects [58]. In acute and severe inflammation, emodin regulates inflammation by regulating the ratios of TH1, TH2, TH17, and *γδ* T cells and regulating the secretion of interferon *γ* and IL-17 from *γδ* T cells [59]. In liver disease, emodin can effectively reduce the expression of proinflammatory cytokines and chemokines in the liver, including TNF-*α*, IFN-*γ*, IL-1*β*, IL-6, IL-12, inducible nitric oxide synthase (iNOS), integrin alpha M, chemokine ligand 2 (CCL2), macrophage inflammatory protein 2 (MIP-2), and chemokine (CXC motif) receptor 2 [60]. However, unlike nonglycosylated emodin, the emodin derivative 8-O-glucoside (E8G) can promote macrophage secretion of the proinflammatory cytokines TNF-*α* and IL-6 by upregulating the TLR-2/MAPK/NF-*κ*B signaling pathway and exerting proinflammatory effects [61].

Emodin can inhibit the expression of CD80 and CD83 in DCs and the secretion of IL-12p70. Emodin-treated DCs exhibit reduced abilities to induce T lymphocyte proliferation and inhibit differentiation and maturation. In addition, emodin can inhibit the secretion of IL-12 by DCs, promote the secretion of IL-10, and inhibit the stimulatory effects of DCS on autologous T lymphocyte proliferation [62, 63]. In addition, physcion, a derivative of emodin, can effectively promote the expression of the DC surface molecules CD40, CD80, CD86, and MHC II, promote the secretion of cytokines by DCs, including IL-12p70, IL-1*β*, IL-6, and TNF-*α*, and induce the maturation of DCs. These effects further promote the differentiation of Th1 cells, do not affect the differentiation of Th2 cells, and effectively improve diseases induced by imbalances in Th1/Th2 cells [63].

In Tregs, emodin can significantly inhibit the expression of human leukocyte antigen (HLA-DR), glucocorticoid-induced tumor necrosis factor receptor (GITR), and cytotoxic T lymphocyte-associated antigen 4 (CTLA-4) and thereby induces Treg maturation and enhances the immunosuppressive function of CD4^+^CD25^+^ Tregs [62]. Emodin can inhibit immune rejection by inducing the maturation of CD4^+^FoxP3^+^ and CD8^+^CD122^+^ Tregs and inhibiting the production of rejection antibodies [64].

These studies show that although emodin can act on multiple immune cells, it ultimately exerts its effects by affecting the secretion of inflammatory cytokines by these immune cells, and inflammatory cytokines are the main pathogenic causes of RA. Therefore, the treatment of inflammatory damage in RA can be achieved by regulating inflammatory cytokines.

## 3. Pathogenesis of RA

Genetic, environmental, and immune activation factors are associated with the pathogenesis of RA. (1) Genetic factors. Heritability of seropositive RA is observed in approximately 40–65% of cases, and seronegative RA is observed in approximately 20% of cases. Genome-wide association studies of single nucleotide polymorphisms have identified more than 100 genetic risk loci associated with RA, and most of these loci are associated with immune mechanisms [1, 5]. The HLA system (particularly HLA-DRB1), as the main influencing factor, promotes the effects of inflammatory and autologous polypeptides on the pathogenesis of RA and thereby exacerbates the inflammatory response. Other genetic loci may play a lesser role, but the effects induced by these loci have cumulative effects that ultimately affect costimulatory pathways, cytokine signaling, lymphocyte receptors, and innate immune activation [6]. (2) Environmental factors. The occurrence of RA is also related to environmental factors. The known risk factors include smoking, low socioeconomic status, and low educational level [65]. It has also been reported that RA is associated with periodontal disease, possibly because *Porphyromonas gingivalis*, a bacterium commonly detected in periodontitis, promotes the endogenous production of recombinant human arginine deiminase 4 (PADI4), which induces abnormal citrulline levels, promotes the conversion of arginine to citrulline, and ultimately reduces tissue tolerance to citrulline peptides [66, 67] (3) Immune activation. The occurrence of RA may also be due to ACPAs forming immune complexes with citrulline-containing antigens. Subsequent binding to rheumatoid factor results in massive complement activation, which promotes the occurrence of an immune cascade. In addition, ACPAs can also be pathogenic by themselves. ACPAs may activate macrophages by binding to antigens to form complexes and then bind to toll-like receptors or Fc receptors to promote inflammatory responses and activate osteoclasts; ACPAs may also bind to citrulline vimentin and promote bone loss. Rheumatoid factor (RF) is more directly involved in the activation of macrophages and cytokines than ACPA [68].

## 4. Inflammatory Cytokines and the Pathology of RA

The pathological changes in RA joints that occur in RA patients include intra-articular and extra-articular changes. The basic pathological change in the joint occurs in synovitis, which manifests as synovial microvascular proliferation. The synovial lining cells proliferate from layers 1–2 to layers 8–10, and the synovial stroma contains a large number of T lymphocytes, plasma cells, and macrophages and shows infiltration of inflammatory cells such as T cells and neutrophils. Based on the above pathology, these cells and blood vessels invade cartilage or bone tissue and form an invasive pannus-cartilage-osseointegration area with obvious cartilage destruction and reduced levels of chondrocytes. The basic pathological changes outside the joints include vasculitis, which mainly manifests as necrotizing full-thickness arteritis of small arteries with mononuclear cell infiltration, intimal proliferation, thrombosis, small veins, and leukocytoclastic vasculitis [1]. The inflammatory cytokines TNF-*α*, IL-6, IL-4, IL-10, IL-13, IL-11, and TGF-*β* play a major dominant role in the pathological changes of synovitis. TNF-*α* is a cytokine with a wide range of effects that can modulate cell proliferation and apoptosis and innate and adaptive immune responses by regulating the NF-*κ*B signaling pathway [69]. IL-6 mainly initiates inflammatory responses through the JAK/STAT signaling pathway, induces the phosphorylation of STAT3 in cells and participates in the activation and proliferation of fibroblasts, osteoclast differentiation, T-cell proliferation and survival, Th17-cell differentiation, B-cell survival, antibody production, and other processes [70, 71]. IL-4 can affect Th-cell differentiation, regulates the polarization and activity of macrophages, and inhibit the production of IL-1*β* and TNF-ɑ by synovial macrophages, and as a result, this cytokine inhibits the development of inflammation [72, 73]. IL-10 activates the JAK1/STAT3 signaling pathway, reduces the release of proinflammatory mediators, and thereby suppresses the immune response [74–79]. IL-13 activates the NF-*κ*B and STAT6 signaling pathways, induces monocyte differentiation, and inhibits inflammatory responses [80–85]. IL-11 acts on the JAK/STAT3 and NF-*κ*B signaling pathways to reduce the production of IL-1 and TNF and thereby reduce the occurrence of inflammation [86]. TGF-*β* can inhibit the proliferation of T lymphocytes and thymocytes and thereby inhibit the immune cascade [87, 88]. The inflammatory cytokines IL-1 and IL-9 act on osteoblasts and osteoclasts during the pathological changes of bone erosion and bone destruction. IL-1 promotes the activation of leukocytes, endothelial cells, chondrocytes, and osteoclasts, and thereby exacerbates RA damage [89]. IL-9 can promote the formation and function of osteoclasts through the M-CSF/sRANKL signaling pathway, which in turn regulates the expression of matrix metalloproteinases (MMPs) and ultimately leads to bone damage in RA [90]. GM-CSF and IL-17 play major regulatory roles in the pathological changes in vasculitis. The synovium in RA patients expresses GM-CSF, and the level of GM-CSF in synovial fluid is increased. GM-CSF plays a key regulatory role in the differentiation, survival, and activation of macrophages and can promote the differentiation of Th17 cells, which ultimately affects the occurrence and development of RA [91–93]. IL-17 can stimulate synovial fibroblasts to produce vascular endothelial growth factor, promote angiogenesis, and increase the number of intra-articular blood vessels, and this cytokine thereby promotes the infiltration of inflammatory cells and their secreted cytokines and exacerbates the inflammatory response [94, 95]. Therefore, during the pathological changes that occur during RA, different inflammatory cytokines cause the different pathological mechanisms of RA.

## 5. Emodin Affects RA Procession by Regulating Inflammatory Cytokines

The immunomodulatory effects of emodin may be partly attributed to its antiproliferative effects on lymphocytes and its regulation of the TH1/TH2 and TH17/Treg balance [96]. To inhibit inflammation, emodin reduces the levels of TNF-ɑ and IL-6 in plasma and inhibits the production of PGE(2), the protein expression of COX-2 in synovial tissue [97] and the synergistic effect of the anti-inflammatory cytokines IL-4, IL-10, IL-13, IL-11 and TGF-*β* outside and inside cells. In the treatment of RA, emodin acts on synovial cells to inhibit inflammation by activating or inhibiting various signaling pathways, such as the JAK/STAT, NF-*κ*B, and OPG/RANK-RANKL pathways (Table 1). In clinical practice, Rt clears heat toxins, regulates intestinal flora and improves the internal environment, and can also reduce the occurrence of RA by regulating intestinal bacteria. Inflammation is a double-edged sword and is essential for host defense [12, 13, 36–38]. In addition, the body's inability to stop the inflammatory response leads to the uncontrolled destruction of cells and tissues and may lead to the development of chronic immune-mediated inflammatory diseases, allergies, or cancer.

Emodin can accelerate the resolution of inflammation by promoting granulocyte apoptosis [131], can significantly alleviate the symptoms of RA in a mouse model by regulating the activity of neutrophils in vivo, and can also reduce the occurrence and development of inflammation by regulating TNF-mediated inflammatory pathways [125, 126]. Emodin may improve symptoms of ulcerative colitis by regulating the flagellin-TLR5 signaling pathway [132]. Emodin induces apoptosis in fibroblasts in patients with ankylosing spondylitis by increasing the levels of active caspase-9, active caspase-3, and Bax and downregulating the expression of Bcl-2 [133]. In the context of allergic reactions, emodin may exhibit antiallergic effects by increasing the stability of cell membranes and inhibiting the source of extracellular calcium [134]. In the context of autoimmune myocarditis in rats, emodin reduces TNF-*α* and IL-1*β* production to reduce inflammatory damage [135].

### 5.1. Proinflammatory Cytokines

In RA, proinflammatory cytokines collectively promote the recruitment of leukocytes in the joints, induce chronic inflammation, stimulate osteoclast formation, induce the proliferation of synovial fibroblasts, lead to pannus formation, promote bone and cartilage degradation, and induce the release of other proinflammatory mediators, and these effects ultimately induce an inflammatory cascade that worsens the pathological changes that occur during RA.

#### 5.1.1. TNF-*α*

TNF-*α* is produced by activated macrophages, monocytes, T cells, and other immune cells and plays a key role in cell proliferation, apoptosis, and innate and adaptive immunity The various biological activities of TNF are mediated by the binding and activation of TNF receptor 1 (TNFR1) and TNF receptor 2 (TNFR2). TNFR1 is widely expressed, whereas TNFR2 expression is restricted to a few specific cell types, mainly including immune cells, endothelial cells, and other synovial cells [136–138]. As a proinflammatory factor, TNF-*α* can induce the proliferation of synovial cells in RA and reduce their apoptosis through the NF-*κ*B signaling pathway Emodin can inhibit the release of TNF from RBL-2H3 cells. In the collagen-induced arthritis (CIA) mouse model, emodin inhibits the levels of TNF-*α* and IL-6 in plasma [97]. Under hypoxic conditions, emodin reduces TNF-*α*, IL-6, IL-8, prostaglandin 2 (PGE2), MMP-1, MMP-13, and VEGF production in lipopolysaccharide (LPS)-induced synovial cells [98]. Emodin inhibits activation of the NF-*κ*B signaling pathway by blocking the degradation of IjBa, directly acts on the NF-*κ*B signaling pathway, and inhibits the degradation of the I*κ*B subunit [99]. Studies have shown that external use of the traditional Chinese medicine compound rhubarb powder exerts a significant effect on relieving joint redness, swelling, heat, and pain in RA patients, and in an RA mouse model, this treatment can reduce the expression of IL-33, MMP-10, TNF-*α,* and other cytokines and increase the level of IL-10 and the ratio of OPG/RANKL, which results in controlling RA inflammation and preventing the exacerbation of disease [100].

#### 5.1.2. IL-6

IL-6 is secreted by monocytes and macrophages following the binding of LPS to Toll-like receptors during infection, inflammation, or cancer [139]. IL-6 exerts biological effects through the IL-6 receptor (IL-6R), which consists of two subunits: a type I cytokine alpha receptor subunit (IL-6R, or CD126) and a common signaling beta receptor subunit (gp130, or CD130) [140]. IL-6 is important for regulating B- and T-cell responses and coordinating the activities of the innate and adaptive immune systems [141]. In RA, IL-6 is highly expressed in serum and synovial tissue and mainly acts through the JAK/STAT signaling pathway to initiate inflammatory responses and induce the phosphorylation of STAT3. Emodin can increase the expression of TUG1 in WI-38 cells through the NF-*κ*B and p38MAPK pathways and thereby reduces LPS-induced inflammatory injury [101]. Emodin also reduces the plasma levels of TNF-*α* and IL-6, PGE(2) production, and cyclooxygenase 2 (COX-2) protein expression in synovial tissue [102].

#### 5.1.3. IL-1

IL-1 is produced by activated macrophages [142], is a key proinflammatory cytokine that affects immune cells, endothelial cells, and numerous target cells in the liver, and is a major causative factor in autoinflammation, autoimmunity, and infection [143, 144]. Its ligands and receptor families are mainly associated with acute and chronic inflammation, and the cytoplasmic fragment of each IL-1 receptor family member contains a Toll-IL-1 receptor domain, which is also present in each Toll-like receptor. In vivo, these receptors respond to microbial products and viruses. One of the 11 members of the IL-1 family, IL-1*β*, has emerged as a therapeutic target for many systemic and local inflammatory diseases (autoinflammatory diseases), which can be treated by reducing IL-1*β* activity to cure acute and chronic inflammatory diseases, and the disease severity is influenced by the anti-inflammatory effects of IL-1 and its receptor [145]. IL-1*β* exerts proinflammatory effects, promotes vasodilation, activates innate immune cells (Neutrophils) [146, 147], and can act on T cells to induce the differentiation of Th17 cells [148]. High levels of IL-1 (IL-1*α* and IL-1*β*) in the synovial membrane and synovial fluid in RA can promote the expression of PGE2 and MMP in fibroblast-like synoviocytes (FLSs) [103, 104]. In a hypoxic environment, emodin can inhibit IL-1*β* and the LPS-induced increased expression of COX-2, VEGF, hypoxia-inducible factor 1*α* (HIF-1*α*), MMP-1, and MMP-13 [98, 105].

#### 5.1.4. IL-17

IL-17 is a proinflammatory cytokine that is mainly secreted by Th17 and other T cells and plays an important role in adaptive immunity. In RA, IL-17 cooperates with TNF to increase the survival of synovial cells and promote their invasion and migration [149, 150]. IL-17 induces the production of G-CSF and CXC chemokine ligands 1 and 2 and thereby promotes the activation of T cells and neutrophils [151, 152]. In an RA model, the intra-articular injection of IL-17 antibodies effectively reduces synovitis symptoms and inhibits bone resorption [106]. The immunomodulatory effect of emodin may inhibit the proliferation of lymphocytes and balance the ratios of Th1 to Th2 cells and Th17 to Tregs. These findings, while providing evidence for the immunomodulatory mechanism of emodin, also have potential implications for promoting the use of emodin to treat RA [69]. In addition, emodin can inhibit viral myocarditis-associated damage by inhibiting the IL-23/IL-17 inflammatory axis, Th17-cell proliferation, and viral replication and thus exerts cardioprotective effects [107].

#### 5.1.5. IL-9

Th9 cells are a newly identified subset of CD4^+^ T cells that secrete IL-9 [153]. rIL-9 stimulation can significantly enhance the secretion of nuclear factor and cytoplasmic 1 (NFATc1) by activated T cells; NFATc1 is a master transcriptional regulator of osteoclast is enhanced differentiation in RA patients in whom the bone resorption capacity of osteoclasts and ultimately induces the differentiation of functional osteoclasts. In RA, IL-9 can lead to bone destruction by promoting osteoclastogenesis and regulating the expression of MMPs. Enhanced formation and function of osteoclasts lead to the disruption of bone homeostasis, which ultimately induces bone destruction [108, 109]. IL-9 levels are elevated in the serum and synovial fluid in RA patients, and a strong correlation has been observed between synovial tissue inflammation and IL-9 levels. The stimulation of IL-9 significantly enhances M-CSF/sRANKL-mediated osteoclast formation and function. Studies have shown that emodin can inhibit the secretion of IL-9 by inhibiting the phosphorylation of IKK and the NF-*κ*B signaling pathway, thereby inhibiting the proliferation of osteoclasts and reducing bone destruction in RA [110].

#### 5.1.6. GM-CSF

GM-CSF is secreted by monocytes, lymphocytes, or fibroblasts and can regulate the differentiation, polarization, and activation of immune cells such as macrophages, DCs, and lymphocytes. GM-CSF is a secreted cytokine that belongs to the colony-stimulating factor family of hematopoietic growth factors and is also a proinflammatory cytokine [154–157]. In RA, the inflammatory changes induced by leukocyte activation can be suppressed using a GM-CSF antibody. The binding of GM-CSF to its receptor can affect downstream signaling molecules, such as JAK2/STAT, mitogen-activated protein kinase (MAPK), NF-*κ*B, and phosphatidylinositol 3 kinase (PI3K), and in turn affect related signal transduction [91, 92, 111–118]. Studies have shown that anthraquinone compounds (emodin methyl ethers) can promote apoptosis in bone marrow cells and osteoclasts induced by GM-CSF and RANKL and promote the expression of osteopontin (OPG) in osteoblasts. In addition, anthraquinone compounds can effectively inhibit the expression of calcitonin receptor (CTR) and carbonic anhydrase/II (CAII) in osteoclasts induced by M-CSF and RANKL by inhibiting the JNK and NF-*κ*B signaling pathways; therefore, anthraquinone compounds have the potential to inhibit bone resorption [119]. In addition, in a CIA mouse model, emodin inhibited macrophage-induced osteoclast differentiation and RANKL expression after M-CSF treatment [120].

### 5.2. Anti-Inflammatory Cytokines

Anti-inflammatory cytokines can neutralize proinflammatory cytokines and suppress both adaptive and innate immune responses. The common anti-inflammatory cytokines in RA are IL-4, IL-10, IL-13, and IL-11, which can balance the ratio between innate and adaptive immune cells [7, 8].

#### 5.2.1. IL-4

IL-4 is secreted by mature Th2 cells, can promote the proliferation of Th2 cells, aid the activation of B cells, and play a role in humoral immunity. IL-4 inhibits the polarization and activity of macrophages induced by proinflammatory cytokines secreted by Th1 cells and enhances Th2 cell-mediated anti-inflammatory effects by regulating histone deacetylation. IL-4 also blocks or inhibits monocyte-derived cytokine secretion, including the secretion of IL-1, TNF a, IL-6, IL-8, and macrophage inflammatory protein (MIP)-1*α*. In RA, IL-4 can inhibit growth factor-induced synovial cell proliferation by interfering with the cell cycle and reducing cell survival and can exert antiangiogenic effects by inhibiting the production of vascular endothelial growth factor in FLSs [158–161]. IL-4, which is an endogenous regulator, inhibits mast cell development and mast cell progenitor survival, reduces the mast cell numbers in a mouse model of CIA and inhibits the production of IL-1*β* and TNF-*α* by synovial macrophages. In addition, IL-4 can inhibit the expression of MMP-13, tissue inhibitor of metalloproteinase 3, or disaggregation protein-like metalloproteinase 4 in chondrocytes. Therefore, IL-4 can inhibit inflammation and prevent bone destruction by regulating the expression of proinflammatory factors, inhibiting the proliferation of synovial cells, and affecting angiogenesis in FLSs [121, 122]. As observed in studies of emodin-regulated macrophages, emodin bidirectionally regulates LPS/IFN-*γ* and IL-4 response genes by inhibiting the NF-*κ*B/IRF5/STAT1 and IRF4/STAT6 signaling pathways and thereby regulates the proliferation, differentiation, and generation of macrophages. As revealed by immunosuppression studies, emodin inhibits IL-2 production and promotes IL-4 secretion in mixed lymphocyte culture medium [123].

#### 5.2.2. IL-10

IL-10 is an immunosuppressive cytokine secreted by T cells, B cells, monocytes, macrophages, neutrophils, and DCs. IL-10 is a potent inhibitor of the expression of Th1-type cytokines (IFN-*γ*, TNF-*α*, and IL-2), attenuates the surface expression of TNF receptors, and promotes the release of TNF receptors into the systemic circulation. The Janus kinase-signal transducer and activator of transcription (JAK-STAT) signaling pathway is a key signaling pathway that mediates the effect of IL-10. IL-10 activates the JAK1/STAT3 signaling pathway after binding to its ligands, initiates specific DNA transcription in the nucleus, and exerts anti-inflammatory effects. In RA, IL-10 inhibits the expression of the proinflammatory factor TNF-ɑ, prevents osteoclast activation, and reduces the degree of joint swelling, and as a result, this cytokine inhibits the progression of inflammation, relieves cartilage degradation, and exerts immunomodulatory effects [69]. In addition, in macrophages in the CIA mouse model, IL-10 deficiency leads to marked upregulation of IL-33 expression and aggravates the progression of CIA in the presence of STAT3 activation; IL-10 deficiency leads to marked upregulation of IL-33 expression and exacerbates the progression of CIA, and treatment with exogenous IL-10 inhibits IL-33 production in IL-10-knockout CIA mice. These results show that IL-33/ST2-mediated inflammation in macrophages is directly abrogated by IL-10 [124].

#### 5.2.3. IL-13

IL-13 is secreted by mature Th2 cells; inhibits the proliferation of Th1 cells; downregulates TNF, IL-1, IL-8, and MIP-1 production by monocytes; upregulates the expression of major histocompatibility complex class II (MHC II) antigens; and activates STAT6 signaling pathway-dependent monocyte differentiation, and this cytokine thereby controls the inflammatory response [69]. In RA, IL-13 can inhibit the production of TNF-*α* by LPS-induced macrophages and reduce the expression levels of various factors, such as the proinflammatory cytokines IL-1*β*, TNF-*α,* and IL-6 in synovial tissue; macrophage inflammatory protein 1*α*; macrophage inflammatory protein 1*β*; and macrophage inflammatory protein 3. IL-13 can also induce the transformation of inflammatory macrophages into anti-inflammatory macrophages, which secrete anti-inflammatory cytokines, such as IL-10 and TGF-*β*. In addition, IL-13 inhibits angiogenesis, synovial cells, and osteoblast apoptosis [125, 126]. In a mouse model of asthma, emodin can stimulate Th2 cells to secrete IL-4, IL-5, and IL-13, which could effectively delay the progression of airway inflammation [127]. Overall, in the RA model, emodin can regulate IL-13 by stimulating Th2 cells.

#### 5.2.4. TGF-*β*

TGF-*β* can be produced by various cells, such as epithelial cells, immune cells, and fibroblasts [162, 163]. TGF-*β* can inhibit the proliferation and differentiation of T cells, B cells, and thymocytes, limit the production of IL-2, IFN-*γ,* and TNF; and increase the secretion of GM-CSF [133, 134, 164–166]. In a mouse model of asthma, TGF-*β* induces the expression of the transcription factor Foxp3 to convert peripheral CD4^+^CD25^−^ naïve T cells into CD4^+^CD25^+^ regulatory T cells and thereby reduces allergic responses in the lungs [167]. In RA, TGF-*β* can enhance the regulatory function of B cells and thus promote the maturation and differentiation of Tregs and restrict the proliferation of T cells and their differentiation into Th1 and Th17 cells [168, 169]. TGF-*β*1 promotes the proliferation of human FLSs [128]. TGF-*β* can act on Th17 cells when combined with IL-6 or IL-21 and thereby inhibits the secretion of IL-17 A/F and TNF-*α* by Th17 cells [129]. Emodin can promote the proliferation and differentiation of Tregs and Th3 secretion [42]. In addition, breast cancer studies have revealed that emodin inhibits TGF-*β*1 secretion by breast cancer cells and macrophages [130].

## 6. Conclusion and Perspective

Inflammatory cytokines play an important role throughout the whole process of RA occurrence and development, and RA can be treated by regulating inflammatory cytokines such as TNF-*α*, IL-6, IL-1*β*, IL-17, IL-4, IL-10, and IL-13. Targeting inflammation in RA is a treatment trend, and the simultaneous regulation of multiple inflammatory cytokines will be of great significance for the treatment of RA. Some cytokine-targeted biologics currently on the market are TNF-*α* receptor inhibitors (etanercept, adalimumab, infliximab, and certolizumab pegol), IL-6 receptor inhibitors (tocilizumab and sarilumab), and IL-1*β* receptor inhibitors (canakinumab), and some of these, such as IL-12 and IL-23 receptor inhibitors, are in the experimental stage. The targeted biological mechanisms of these cytokine receptors exert substantial anti-inflammatory and bone protection effects in RA [7, 8], but caution is needed when biological agents are used in patients with low white blood cell counts, liver and kidney insufficiency, *tuberculosis,* and hepatitis B. In addition, the long-term use of biologics can lead to many serious adverse events, particularly infections and allergic reactions, which can increase the pressure and financial burden on patients and also cause mental and physical trauma to patients. Therefore, the identification of a reasonable, safe, and effective drug is important for the treatment of RA [170].

Emodin is a natural anthraquinone compound with various pharmacological effects, including anticancer, anti-inflammatory, antiviral, antibacterial, antiallergic, antiosteoporosis, antidiabetic, immunosuppressive, neuroprotective, and hepatoprotective effects. This compound has low immunogenicity and exerts strong anti-inflammatory effects; the main metabolic pathways are glucuronidation and sulfonation metabolism; emodin also exhibits high bioavailability and exerts a protective effect on patients with renal insufficiency. Regarding inflammatory cytokines, emodin further regulates various inflammatory diseases by regulating the secretion of cytokines and has no toxic side effects during the entire treatment process. Emodin, as an extract of a monomer used in traditional Chinese medicine, has many benefits and a low price and is easily accepted by the majority of patients (Figure 4).

Inflammatory cytokines are the most direct factors that lead to the occurrence and development of RA. The direct regulation of these cytokines is of great value to the treatment of RA. The simultaneous regulation of multiple inflammatory cytokines will be beneficial for the treatment of RA. However, recent studies have shown that the simultaneous use of two inflammatory cell-targeting biological agents in the treatment of RA increases the risk of infection in patients and has obvious side effects. As discussed in this review, emodin acts synergistically on proinflammatory and anti-inflammatory cytokines through multiple signaling pathways and has the potential to inhibit inflammatory damage in various diseases. Controlling inflammation will control the progression of RA, but the treatment of RA is not limited to directly inhibiting inflammation, and balancing the relationship between proinflammatory and anti-inflammatory cytokines will become a future direction of research on RA treatment. Emodin acts on a variety of proinflammatory cytokines and anti-inflammatory cytokines at the same time, and the effect is considerable. This review provides a reference for further combined drug treatment for RA in the future and is worthy of clinical application.

## Figures and Tables

**Figure 1:** (a) Traditional Chinese medicine RHEI RADIX ET RHIZOMA. (b) Chemical structure and molecular weight of emodin. (c) The number of articles published on emodin each year over the past 20 years has increased each year.

**Figure 2:** In human diseases, Emodin has a variety of biological regulatory functions, such as immunoregulation, antivirus, anticancer, antioxidant, proliferation regulation, and kinase regulation. Therefore, emodin has therapeutic potential in diseases of the cardiovascular system, respiratory system, metabolic system, nervous system, and other systems.

**Figure 3:** In immune cells, emodin can induce T-cell apoptosis, inhibit the expression of Tregs, and inhibit macrophage polarization. Therefore, emodin can regulate these immune cells to control the inflammatory reaction and inflammatory cytokines.

**Figure 4:** In RA, emodin can promote the secretion of anti-inflammatory cytokines (IL-4, IL-10, IL-13, and TGF-*β*) and inhibit the secretion of proinflammatory cytokines (TNF-*α*, GM-CSF, IL-6, IL-1, IL-17, and IL-9), through the different signal pathways to reduce the inflammatory reaction and regulate the osteoblasts and osteoclasts to relieve the bone erosion and destruction.

**Table 1:** The regulatory mechanism of emodin in inflammatory cytokines in RA.

Species	Inflammatory cytokines	Target	Regulation results	Refs.
Proinflammatory cytokines	TNF-*α*	NF-*κ*B	TNFa, IL-6, IL-1*β*, IL-6, IL-33, MMP-10, and IL-8 decreased expression	[97–100]
	IL-6	PI3K/AKT	TNF-*α*, IL-6, PGE (2), and COX-2 decreased expression	[101, 102]
	IL-1, IL-1*β*	FPGE2, C'ase	PGE2, MMP-3, MMP-13, ADAMTS-4, and ADAMTS-5 decreased expression	[98, 103–105]
	IL-17	G-CSF, CXC chemokine ligands 1 and 2	Balance the ratio of TH1/TH2 cells and TH17/Tregs	[69, 106, 107]
	IL-9	M-CSF/sRANKL	Inhibiting the phosphorylation of IKK and RANKL expression	[108–110]
	M-CSF	JAK2/STAT5	Enhances RANKL-dependent apoptosis of osteoclasts	[92, 111–120]

Anti-inflammatory cytokines	IL-4	MMP-13, metalloproteinase 3, and protein-like metalloproteinase 4	Inhibiting the NF-*κ*B/IRF5/STAT1 and IRF4/STAT6 signaling pathways, Inhibiting M1-to-M2 polarization of macrophages	[75, 121–123]
	IL-10	JAK1/STAT3	Inhibiting the PI3K/AKT signaling pathways, inducing DC maturation, and promoting Th1 cell polarization	[124]
	IL-13	STAT6	IL-1*β*, TNF-*α*, IL-6, macrophage inflammatory protein 1*α*, macrophage inflammatory protein 1*β,* and macrophage inflammatory protein 3 decreased expression	[125–127]
	TGF-*β*	T cells, B cells, and thymocytes	Inhibiting the proliferation and differentiation of T cells, B cells, and thymocytes, limit the production of IL-2, IFN-*γ,* and TNF, and increase the secretion of GM-CSF	[42, 128–130]

## Data Availability

Not declared.
